# The Oral Tumor Cell Exosome miR-10b Stimulates Cell Invasion and Relocation via AKT Signaling

**DOI:** 10.1155/2022/3188992

**Published:** 2022-08-16

**Authors:** Xiang Li, Ting Yang, Chuanji Shu

**Affiliations:** ^1^Department of Stomatology, Huangshi Central Hospital, Affiliated Hospital of Hubei Polytechnic University, Edong Healthcare Group, Huangshi 435000, China; ^2^Department of Dermatology, Huangshi Central Hospital, Affiliated Hospital of Hubei Polytechnic University, Edong Healthcare Group, Huangshi 435000, China

## Abstract

An exosome derived from a cancer cell has been identified to regulate intercellular communication. However, the roles of oral cancer-derived ectodomains in tumor metastasis need to be investigated further. We investigated their roles in oral cancer cells in this paper. The enforcing effect on oral cancer cells was attributed primarily to miR-10b, a gene with a high level in exosomes that is transferred to recipient cells via oral cancer-derived exosomes. Exosomes were obtained by exosome isolation reagents. Also, exosome identification and analysis were performed by electron microscopy. The expression of miRNAs was analyzed by qRT-PCR. Protein expression was analyzed by Western blot. Also, invasion and migration experiments were performed to assay and evaluate the function of exosomal miR-10b. Exosome-mediated transfer of miR-10b promoted oral cancer cell behaviors, according to the findings. Finally, it was discovered that AKT signaling participates in regulating exosome-mediated invasion and migration of oral cancer cells and its activation reduced the inhibitory effect of miR-10b knockdown on oral cancer cells. Exosomal miR-10b derived from oral cancer cells enhances cell invasion and migration by activating AKT signaling.

## 1. Introduction

Oral cancer is a common prevailing cancer with high mortality [1]. Oral cancer has a strong migration and invasion ability, and metastasis is one of the main reasons for patients' poor prognosis. As a result, it is critical to understand the mechanism of oral cancer metastasis in order to improve patient prognosis.

Exosomes are secreted by cells and serve as a vital modulators in many processes. The function of exosomes in cancer development has been well identified. Exosomes containing Wnt4 are, for example, secreted by colorectal cancer cells in a hypoxic environment and transferred to normoxic cells to promote proliferation and invasion [2]. Exosomal CLIC1 regulates vincristine resistance to gastric cancer [3]. Moreover, many studies showed the critical role of exosomes in cancer cell invasion and migration. For example, exosomal LOXL4 facilitates hepatocellular carcinoma cell invasion and metastasis [4], and exosomal thrombospondin 1 is involved in lung cancer migration and invasion [5]. Exosome THBS1 enhances malignant migration of oral squamous cell carcinoma via M1 macrophage activation [6].

MicroRNAs, a class of 18–23 nucleotide noncoding RNAs, can be transferred by exosomes and function in cancer development [7]. In gastric cancer, exosomal miR-1290 promotes cell proliferation [8]. Exosome-mediated miR-21 enhances cell invasion in esophageal cancer [9]. Macrophage-derived exosome miR-92a-2-5p promotes liver cancer cell invasion [10]. miR-10b is a crucial miRNA and is significantly involved in the regulation of cancer regulation including oral cancer. It was found that miR-10b may affect the early detection of oral cancer [11]. Most importantly, miR-10b can serve as an exosome and derive the cancer metastasis, and its transfer mediated by the exosome can enhance breast cancer cell invasion [12]. Acidic-regulated increased exosomal miR-10b promotes hepatocellular cancer metastasis [13]. However, its role in oral cancer is unclear. Our study aims to investigate its role in oral cancer cells.

## 2. Materials and Methods

### 2.1. Cell Culture

Oral cancer cell lines HSC-6 and THP-1 were purchased from Chinese Academy of Sciences (Shanghai, China). HSC-6 and THP-1 were cultured in a medium containing 100 *μ*g/mL streptomycin, 100 U/mL penicillin (Hyclone Laboratories, Inc), and 10% fetal bovine serum (Gibco, Carlsbad, CA, USA) in DMEM (Hyclone Laboratories, Inc., Logan, UT, USA) and cultured in a constant temperature cell incubator (37°C, CO_2_ volume fraction 5%).

### 2.2. Cell Transfection

HSC-6 cells were transfected with miR-10b inhibitor and NC (GenePharma) using Lipofectamine 2000 reagent (Invitrogen, USA). The transfection was measured by RT-qPCR.

### 2.3. Exosome Isolation

Exosomes were obtained from HSC-6 cells by Ribo™ Exosome Isolation Reagent (RiboBio, C10130-1) according to the instruction and identified by scanning electron microscopy.

### 2.4. Exosome Uptake

Exosomes isolated from oral cancer cells were labeled with PKH67 dye, and DAPI was used for nuclear staining. After incubation, exosome uptake was examined by confocal microscopy.

### 2.5. Invasion and Migration Assay

Evaluate cell invasion and migration. HSC-6 cells (2 × 10^4^ cells per well) were seeded in the upper chamber of the Transwell, serum-free culture medium was placed in the lower chamber, and SDF-1 was added to the culture medium. HSC-6 cells were removed after 12 hours of incubation, cleaned, fixed, crystallized, and quantified using Image Pro Plus.

### 2.6. Western Blot

Cellular proteins were isolated using RIPA buffer, and proteins were then denatured by boiling. The total concentration of protein was determined by a bicinchoninic acid assay (Beyotime Institute of Biotechnology). The protein was separated using electrophoresis at 90 V for 100 min and then transferred to a nitrocellulose membrane at 110 V for 75 min. The membrane was blocked with skimmed milk for 2 h and then incubated with the following antibodies: anti-AKT (1 : 1000; AA326; Beyotime), anti-p-AKT (1 : 1000; AA329; Beyotime), and anti-GAPDH (1 : 5000; 10494-1-AP; Proteintech). Shake on a decolorization shaker at 4°C. Subsequently, we washed the membranes (three times for 15 min, each wash) with TBST and incubated them with goat anti-rabbit (1 : 3,000, Abcam, Cambridge, MA, USA) for 2 h at 26 ± 2°C. Afterward, the membranes were rinsed with TBST (three times/15 min each). We then visualized Western blot bands using the ECL detection system (Bio-Rad).

### 2.7. qRT-PCR

Total RNA was isolated and reversely transcribed to cDNA followed by real-time (RT)-PCR using SYBR Green Master Mix (Biosharp; BL705A). Gene level was analyzed using the ΔΔCt quantification method. The primers were U6 sense 5′-CTCGCTTCGGCAGCACA-3′, U6 antisense 5′- AACGCTTCACGAATT TGCGT-3, miR-10b sense 5′- ACACTCCAGCTGGGTACCCTGTAGATCC -3′, and miR-10b antisense 5′- CTCAACTGGTGTCGTGGA-3.

### 2.8. Statistical Method

All data analyses were conducted using IBM SPSS Statistics for Windows, version 27.0 (IBM Corporation, Armonk, NY, USA). The Western blots were placed into ImageJ for analysis. Plots were generated using Prism 8.0 software (GraphPad Software, Inc., San Diego, CA, USA). The data are presented as mean ± standard deviation, as determined by one-way variance analysis with Tukey's test. *P* < 0.05 was considered statistically significant.

## 3. Results

### 3.1. Characterization of Exosomes from Oral Cancer Cells

The exosomes were obtained by Ribo™ Exosome Isolation Reagent. To identify exosomes, we performed electron microscopy assays.  Figure1 demonstrates the characterization of exosomes secreted by oral cancer cells. As shown in Figure 1(a), the specific exosome morphology and size were about 100 nm in diameter. To further determine the maturity of oral cancer cell-derived exosomes, we next measured the exosome-specific makers including CD63, Arg-1, and TGS101 by Western blotting. The expression of CD63, Arg-1, and TGS101 was higher in exosomes than in cell lysate, as shown in Figure 1(b).

### 3.2. High miR-10b in Exosomes from Oral Cancer Cells

We then determine whether exosomes can be internalized by oral cancer cells, and exosomes were labeled with PKH67 dye (Green).  Figure 2 shows a high miR-10b level in exosomes from oral cancer cells. The uptake of exosomes was visualized under a confocal microscope, as shown in Figure 2(a). A number of studies reported the role of cancer cell-derived miR-10b in cancer development [14], and we next measured its role in oral cancer and found significantly upregulated miR-10b in exosomes from oral cancer cells, as shown in Figure 2(b).

### 3.3. miR-10b Is Transferred to Recipient Cells by Exosomes

Figure 3 shows that miR-10b was transferred to recipient cells by exosomes and promoted oral cancer cell invasion and migration. Exosome administration increased miR-10b expression, as shown in Figure 3(a), and promoted oral cancer cell invasion and migration, as shown in Figure 3(b).

### 3.4. Inhibition of miR-10b Attenuates Oral Cancer Cell Behaviors

We next reduced miR-10b expression in an oral cancer cell by transfection of miR-10b inhibitor and found decreased miR-10b expression after inhibitor treatment, as shown in Figures 4(a) and 4(b). mir-10b that inhibits exosome secretion and nonsense inhibitors were used to coculture with oral cancer cells, and it was found that mir-10b significantly decreased in oral cancer cells when mir-10b secreted by exosomes was inhibited, as shown in Figure 4(c). More importantly, transwell assays showed that incubation with miR-10b inhibitor exosomes attenuated oral cancer cell invasion and migration, as shown in Figure 4(d). The data suggested that oral cancer cell-derived exosomal miR-10b could enhance oral cancer cell invasion and migration.

### 3.5. Exosomal miR-10b Promotes Oral Cancer Cell Behaviors via AKT Signaling

miR-10b is involved in AKT signaling activation [15]. In addition, AKT contributed to the malignant potential of oral cancer [16, 17]. Thus, we sought to explore whether exosomal miR-10b regulates oral cancer cells via activating AKT signaling.  Figure 5 shows that exosomal miR-10b promotes oral cancer cell behaviors via AKT signaling. The expression of phosphorylated AKT was significantly increased after oral cancer cell-derived exosome treatment; however, inhibition of miR-10b reduced phosphorylated AKT level, as shown in Figure 5(a). We next treated exosomes incubated oral cancer cells with AKT activator, SC79, as shown in Figure 5(b). The protein expressions of AKT and p-Akt in exosome-cultured oral cancer cells treated with AKT activator (SC79) were significantly higher than those in exosome cultured oral cancer cells, as shown in Figure 5(c). The data indicated that exosomal miR-10b promoted oral cancer cell behaviors via activating AKT.

## 4. Discussion

Several studies indicated that exosomes derived from cancer cells participate in cancer progression, such as malignant melanoma [18], lung cancer [19], and pancreatic cancer [20]. Of note, exosomes carrying miRNAs are important to tumorigenesis [21].

It is well known that exosomes contribute to oral cancer angiogenesis [22] and regulate natural killer cells and tumor immunity [23]. In addition, exosomes containing miRNAs are also involved in oral cancer progression. Exosomal miR-21 from hypoxic oral squamous cell carcinoma cells promotes prometastatic behaviors of tumor cells [24]. miR-10b has exosome-mediated cancer cell malignant properties. Qian et al. demonstrated that miR-10b-5p was delivered by hypoxic glioma exosomes to normoxic glioma cells to affect cell behaviors [25]. Singh et al. showed that exosomal miR-10b promotes breast cancer cell invasion [12]. Of note, miR-10b is upregulated in oral cancer [11]. Our study found an increased miR-10b level in oral cancer cell-derived exosomes and it could be transferred to the oral cancer cell. The administration of exosomal miR-10b promotes cancer cell behaviors, which were impaired by miR-10b inhibition, indicating that exosomal miR-10b contributes to the progression of oral cancer.

miRNAs exert effects through modulating downstream targets or different signaling pathways. Numerous targets of miR-10b and their role in cancer development have been reported, such as hyaluronan synthase 3 (HAS3) in prostate cancer [26] and phosphatase and tensin homolog (PTEN) in colorectal cancer [27]. In addition, accumulating evidence indicated that miR-10b modulates cancer cell malignancy via AKT signaling. For example, miR-10b regulates breast cancer stem cells via activating AKT [28]. miR-10b attenuates radiosensitivity of glioblastoma cells via AKT [29]. miR-10b facilitates gastric cancer cell invasion. Thus, we sought to explore whether exosomal miR-10b affects oral cancer cells. The results reveal that oral cancer cell-derived exosomal miR-10b can enhance AKT signaling. Moreover, inhibition of miR-10b decreases reduced phosphorylated AKT level and activation of AKT signaling could recover the inhibitory effect of miR-10b knockdown. mir-10b secreted by exosomes can increase the invasion and migration of oral cancer cells by regulating the AKT signaling pathway.

## 5. Conclusions

Exosomes derived from oral cancer cells promote cancer cell invasion and migration. The forced effect on cell invasion and migration is mainly attributed to miR-10b, which is transferred to recipient cells by oral cancer-derived exosomes. The experimental results show that miR-10b transfer mediated by exosome facilitates oral cancer cell invasion and migration by activating AKT signaling. In our future work, the new function of oral cancer-derived exosomes in regulating oral cancer invasion and migration will be explored in depth.

## Figures and Tables

**Figure 1:** Characterization of exosomes secreted by oral cancer cells. (a) Exosomes isolated from HSC-6 cell were assessed by microscopy. (b) Expressions of exosome markers were detected by Western blot.

**Figure 2:** miR-10b level in exosomes. (a) Cellular uptake of exosomes by confocal microscopy. (b) miR-10b level in HSC cell-derived exosomes (^*∗*^*P* < 0.05 (mean ± SD, *n* = 3)).

**Figure 3:** miR-10b is transferred to recipient cells and promotes oral cancer cell invasion and migration. (a) miR-10b level in exosome-treated HSC-6 cell was measured by RT-qPCR assay. PBS-treated HSC-6 cell was used as control (^*∗∗*^*P* < 0.01). (b) Cell invasion and migration (^*∗∗*^*P* < 0.01 (mean ± SD, *n* = 3)).

**Figure 4:** Inhibition of miR-10b attenuates oral cancer cell invasion and migration. (a) miR-10b expression in HSC-6 cell with NC inhibitor exosome or miR-10b inhibitor exosome administration was measured by RT-qPCR assay (^*∗∗∗*^*P* < 0.0001). (b) miR-10b level in NC inhibitor or miR-10b inhibitor-transfected HSC-6 cells was detected by RT-qPCR assay (^*∗∗∗*^*P* < 0.001). (c) miR-10b expression (^*∗*^*P* < 0.05). (d) The invasion and migration of HSC-6 cell with NC inhibitor exosome or miR-10b inhibitor exosome administration (^*∗∗*^*P* < 0.01; ^*∗∗∗*^*P* < 0.001).

**Figure 5:** Exosomal miR-10b promotes oral cancer cell behaviors via AKT signaling. (a) AKT and p-AKT levels in HSC-6 cell with PBS or NC inhibitor exosome or miR-10b inhibitor exosome treatment. (b) AKT and p-AKT levels in HSC-6 cell. (c) The invasion and migration of HSC-6 cell (^*∗*^*P* < 0.05, ^*∗∗*^*P* < 0.01, and ^*∗∗∗*^*P* < 0.001).

## Data Availability

The simulation experiment data used to support the findings of this study are available from the corresponding author upon request.
